RETRACTED

# Big Data Enabled the Development of Public Sports Health Emergency Corpus: Taking MACPHE as an Example

**DOI:** 10.1155/2022/8717072

**Published:** 2022-09-10

**Authors:** Hongjing Cui, Huican Zhang, Deng Pan, Bing Zhao

**Affiliations:** ^1^School of Foreign Languages, Harbin University, Harbin 150086, China; ^2^College of Urban and Environmental Sciences, Central China Normal University, Wuhan 430079, China; ^3^School of Foreign Languages, Hubei University of Science and Technology, Xianning 437100, China; ^4^School of Humanities, Huzhou University, Huzhou, 313000, China; ^5^Philippine Christian University Center for International Education, Manila 1004, Philippines

## Abstract

This study aims to make public sports health emergency corpus as a way to deal with public health emergency such as COVID-19, reducing the losses affected by an illness or health condition that has occurred frequently in recent years. On this basis, this paper analyzes the research status of emergency language services at home and abroad, discusses the significance and principles of Multimodal Aligned Corpus Public Health Emergency (shorted for MACPHE) construction, and develops technical processing paths and building procedures for MACPHE. Finally, it was emphasized that the construction of MACPHE and emergency language resources are important parts of the national language service capacity. Furthermore, on the basis of big data, a modal architecture of MACPHE was given and analyzed in the field of public health service.

## 1. Introduction

Recent public health emergencies, such as COVID-19, Yellow Fever (2016), and Ebola virus disease (2014-15), and outbreak around the world, have highlighted major challenges and gaps in how risk is communicated during epidemics and other health emergencies. Due to the challenges of different social, economic, political, and cultural factors, it influences how people access and trust health information. Furthermore, it will affect people's perception of public health emergencies risk and their risk-reduction behaviors.

Language is one of the vital factors to human daily activities of communication and organization. The role of language is to achieve the function of communication and empathy, which is especially important in the handling of major emergencies. When natural disasters, accidents, and other emergencies occur, use language (including text and spoken), body languages, language technology, language standards, language data, language products, and language-related derivatives to participate in emergency actions and processes to avoid deterioration of the situation and expansion of the situation. We can classify emergency languages into the emergent incidents according to different criteria. For example, from the perspective of language factors, it can be divided into foreign language emergency, minority language emergency, dialect emergency, and mother tongue emergency (such as language public opinion guidance and collection). Therefore, in the process of dealing with major public health emergencies, constructing the multilingual and multimodal public health corpus is very important.

RETRACTED

Emergency language ability originated from the strategic concept of national language ability [1]. They believed that there is a potential need, current demand, and supply in the American language which does not match the national language ability [2]. After that, emergency language ability defined the national language ability in relative detail from the perspectives of talent training sector and language field [3]. The research institutions of language proficiency in the United States include teaching and research institutions, the federal government, private institutions, language inheritance institutions, and overseas institutions. They also defined language proficiency as the sum of different language domains, including the basic system for determining language proficiency, teaching support systems and mechanisms, and high-quality high-level language teaching. Some scholars delineated the global language strategy of the United States; the global strategy discussion covers three parts: the country's foreign language ability needs, the state-led foreign language project cluster, and foreign language projects and their effectiveness [4]. This problem-driven research suggests establishing a national language learning framework to build national language capabilities by improving the national language capabilities of the nationals. Subsequently, some American scholars carried out related research cases, such as [2–6]. This group of scholars clearly pointed out the essential elements of national language ability and the scope of application in public health emergencies.

The concept of emergency language services was first introduced to China by Prof. Li., who defined that the main body that exercises national language ability is the governmental responsibility [7]. The territory where language ability is exercised covers both domestic and foreign countries. The time to exercise language ability spans the present and future. Language proficiency is a kind of language proficiency, including five aspects:(1) language proficiency; (2) national and international status of major languages; (3) citizen language proficiency; (4) ability to possess modern language technology; (5) national language life management level. Later, some scholars commented and discussed it. During the first decade of 21^st^ century, some scholars, such as [8–11], had a clear discussion on its extension and connotation of emergency language services.

RETRACTED

Multimodal corpora, an integration of audial, visual, and textual records, provides a platform to explore the meaning expressed in multimodal discourse. Multimodal corpora can be defined as the digitized collections of language and communication-related material, drawing on more than one modality. That means multimodal corpora involves not only texts but other sensory modalities (i.e., sight, hearing, touch, smell, or taste) or production modalities (i.e., gesture, speech, touch, smell, or taste). According to Allwood's definition in a narrow sense, it is required that transcriptions and annotations should accompany the material in the corpus. Such a definition reveals the nature of the collected material, containing recordings, annotations, and transcriptions. For example, a multimodal corpus may be an integration of texts illustrated with pictures and diagrams or a collection of films annotated with transcriptions of the actors' talk and gestures in the films. The most common multimodal corpora are digitized collections of audio-recorded and video-recorded material of human communication annotated with transcriptions of talk or gestures in the recordings. The modalities embodied in the corpora are, thus, vision and hearing. Multimodal corpus analysis is a corpus-based study combined with systemic functional linguistics and semiotics to testify meaning-making hypotheses in multimodal discourses [9].

International Conference on Language Resources and Evaluation, shorted for LREC as the top conference supported by UNESCO, released the latest academic product about multimodal corpus every two year. We can summarize the general picture of multimodal database from its website (http://lrec-conf.org/). From 1998 to 2021, European Language Resources Association votes for the most important multimodal data projects, such as ISLE, INE, SIMILAR, CHIL, AMI, VACE, and CALLAS [12].

Similar to traditional monolingual corpora, the contents of multimodal corpora, the ways in which they are recorded, and their size are highly dependent on the aims and objectives, specific research questions, and technological or methodological questions of the research project [13]. Given this, there are various types of multimodal corpora related to different research purposes, all of which are customized with a set of characteristics regarding design and infrastructure, size and scope, naturalness, availability, and (re)usability.

The innovations of this paper are mainly reflected in the following aspects: (1) public health emergencies have frequently occurred in recent years, which seriously threaten social stability and the safety of people's lives and property. Based on this, the research content is of great social practical significance and practical value; (2) this article uses the power of big data technology to propose that data-driven technology is embedded in the construction of public health emergencies corpus, which has certain practical results; (3) this articles not only rely on the text corpus but also employed multilingual and multimodal corpus to construct a small-scale aligned corpus to respond to and resolve public health emergencies.

RETRACTED

## 2. Literature Review

### 2.1. Public Health Emergency Research

Research on emergency language services in China has only started in the present decade. In 2012, Chinese National Language Commission (NLC) promulgated the outline of the National Medium and Long-Term Language and Character Reform and Development Plan (2012-2020), which will directly formulate language policies for responding to international affairs and emergencies, raising it to the height of national security. Thirteenth Five-Year Development Plan for Chinese Language and Characters (2016) made it more significant that we should actively establish an effective precaution and emergency response mechanism for language problems and emergencies and strive to improve the national language service response ability. No matter from the perspective of national strategy or national policy, a long-term emergency language service system should be established. Tong pointed out that language service work in an emergency situation is one of the important indicators for testing the language ability of the country [14]. Wang proposed that emergency language ability is an important manifestation of the modernization of social governance capabilities [15]. However, at present, there is still insufficient theoretical research on the language emergency response capabilities of emergencies, inadequate organizational systems, incomplete personnel reserves, inadequate language technology, language resource construction, and practical experience, which cannot fully meet the needs of national development. Especially cannot meet the needs of dealing with emergencies.

In western countries, public health emergency gained a lot of governments' attention since the era of 21^st^ century. The language response mechanism, speed, and effect in the handling of emergencies reflect the level of crisis governance. Emergency language ability may include emergency foreign language (especially non-universal language) ability, emergency dialect ability, industry or field emergency language ability, network emergency language ability, emergency discourse communication ability, and emergency sign language ability. The role of emergency language ability in public emergencies should be played from the following five aspects: one is to improve the emergency language awareness of the whole society, the second is to establish an emergency language response mechanism, the third is to use emergency language talents, and the fourth is to increase technology. Fifth, the application of emergency language service is to strengthen emergency dissemination.

RETRACTED

The application research on the level of emergency language services focuses more on how language technology is used in disaster first aid and management [16]. The following three aspects are mainly discussed:

Firstly, the negative consequences caused by the failure of crisis communication. The fact has been found that in the evacuation of the tsunami and shooting incidents, the use of English alone would cause misunderstandings by English-speaking students; Hispanic workers made the wrong decision because of insufficient understanding of the severity of the disaster [17].

The second issue is the important role of translation and machine translation technology in disaster information release and early warning. From a study of hurricane disaster in the US, because 72.8% of the local residents' mother tongue was not English, local emergency departments encountered huge language barriers when issuing disaster warnings, and local professional translation agencies were also affected by the hurricane, unable to provide language services, thus increasing the difficulty of disaster communication. Some related research topics focused on the disaster trust reconstruction [17]; another research showed interest on the use of disaster translation technology and emergency translation talent training [17]. Through interviews with Japanese disaster survivors that the translation was used in earthquake news broadcasting, nuclear Government disaster emergency response procedures played an important role; he studied how Japan used text-to-speech technology to deal with earthquakes when hosting the Olympic Games [18]. From availability, accessibility, and acceptability of these four dimensions of adaptability (4As), some researchers surveyed the disaster emergency translation measures taken at the national level in Ireland, Japan, New Zealand, the United Kingdom, and the United States; the language technology mainly used in emergency disaster management includes the translation memory technology for handling critical information in disaster emergency. He claimed to ensure that the terminology is always uniform and clear, used to grab life's terminology management technology, online translation management platform technology for managing emergency volunteer translations, and Microsoft's Skype translation technology (real-time conversion of voice information and text information through machine translation in case of emergency and wearable voice machine translation technology, to help patients deal with emergencies) [19].

RETRACTED

The third is the application of emergency language services after the disaster. Chinese scholar surveyed 113 language service companies across the country and found that the new coronavirus pneumonia epidemic has affected the language service industry to varying degrees [15]. On the one hand, companies generally reflect that the language service industry will face downward pressure, and the on-site business of language services will plummet. Nearly 80% of companies are worried about the decline in performance. Most companies hope that the government will reduce taxes or provide subsidies. On the other hand, language service companies strive to save themselves. Online working resume over 90%, language service companies actively participate in combating the epidemic.

### 2.2. Standard Model of Public Health Emergency

#### 2.2.1. Standardization of Emergency Language Services

Research on emergency management standardization was issued in 2004, and the ISO/TC223 Public Safety Standardization Technical Committee came into being international standardization of emergency management in 2004, studying and formulating international standards for public safety management systems; ISO/TC 292 Safety and Resilience Technical Committee was established in 2014 to replace the ISO/TC 223 committee and formulate international safety-related standards from a broader perspective [20].

Because emergency management requirements are highly relevant to national legislation, international standards for emergency management only contain guidelines rather than requirements. The ISO/TC 292 Technical Committee has currently released 8 international standards for emergency management, including incident management guidelines, public warning guidelines, color-coded alert guidelines, capability assessment guidelines, guidelines for monitoring facilities by confirmed hazard levels, and community efficient early warning system implementation guidelines, information interaction structure, exercise guide, and social media application guide.

#### 2.2.2. Significance of Public Health Emergency Corpus Construction

Corpus is a corpus warehouse or a collection of language materials. Emergency corpus refers to a collection of professional language materials with a certain structure, representativeness, and a certain scale, which are specially collected for natural disasters or public crisis events.

1. Building an emergency corpus is an important data foundation for providing rapid rescue language products, language technology, or participating in language rescue operations, including disaster relief language software development, disaster relief language resource management, emergency language standard development, first aid language training, language therapy and rehabilitation, language consultation, and crisis intervention. Emergency language service is an important part of language service. It is a complete system in itself, covering many aspects such as emergency language infrastructure, emergency language planning, emergency language standards, emergency language ability, emergency language talents, and emergency language disciplines. The emergency corpus is the data cornerstone of the complete system of emergency language services
2. Build an open general emergency corpus and terminology knowledge base. By building an open source platform to collect, process, and upgrade information resources related to emergencies, establish a professional and standardized terminology database of Chinese and dialect pairs, sign language symbols, etc. to ensure emergencies. Non-commercial language resource sharing platform where event information data can be exchanged in real time with a unified standard
3. Constructing an emergency corpus can be used to study the language features of Internet texts of major emergencies, reveal the macro and micro models of the dissemination of network information of major emergencies, distinguish the authenticity of network emergencies, and explore the mood swings of netizens in special situations And in the group characteristics of the audience in different contexts, it is of great significance to provide scientific emergency measures and prevention plans for the government and relevant departments

In this article, we propose an architecture of emergency corpus for public health emergency. Regarding the classification of emergency corpora, there is currently no unified standard. We adopted the “General Emergency Response Plan for National Public Emergencies” system, which is issued by the State Council on January 8, 2006. The proposed information processing-oriented emergency corpus classification system includes two levels. Namely, level1 includes 4 categories, and level2 includes 33 subcategories. The specific classification is as follows:

1. Natural disaster N (Natural disaster). It mainly includes 8 subcategories: flood and drought disasters, meteorological disasters, earthquake disasters, geological disasters, marine disasters, biological disasters, forest and grassland fires, and cosmic disasters
2. Accidental emergencies (Accident). It mainly includes war and violence, industrial and mining business safety accidents, transportation safety accidents, urban lifeline accidents, communication safety accidents, environmental pollution and ecological damage, serious fires, poisoning incidents, and acute chemistry. There are 13 subcategories including accidents, radio-logical accidents, medical accidents, expeditionary deaths, and tourism accidents
3. Public health events (Public health). It mainly includes 5 subcategories: epidemic situation of infectious diseases, diseases of unexplained groups, food safety and occupational hazards, animal epidemic situations, other events that seriously affect public health and life safety
4. Social security incidents(Social safety). It mainly includes terrorist attacks, major criminal cases, economic security incidents, foreign-related emergencies, large-scale mass incidents, ethnic religions, anti-government, and anti-socialism 7 subcategories such as riots. Since the limited length of the article, we only present the 2 levels and 4 categories of level 1, and 27 categories of level 2 are shown in Figure 1

RETRACTED

## 3. Methodology: Model Setting of Public Health Emergency Corpus

### 3.1. Big Data Enabled Obtaining Raw Data

There are three main sources of corpus: first, the relevant national laws and regulations text. Secondly, due to the suddenness, contingency, and unpredictability of emergencies, related news web pages and blogs have the advantage of responding faster than other traditional media, so the Internet is one of the best sources for collecting public health emergencies data. Thirdly, social media as the most flexible and interchangeable media gains lots of attention by young people, which can carry profound latest public health emergency news. We mainly use the following two methods to collect emergency news resources from the Internet. That is: (1) using search engines to collect resources; (2) using existing news websites to collect resources. In order to prevent the mutation of information in the process of dissemination, we do not include all reprinted news and self-media articles. Thirdly, we can download some reports from global official website, such as World Health Organization (https://openwho.org/) [21].

The application of artificial intelligence technology to the response and handling of major public health emergencies proposed in this article mainly involves big data technology controlling the official and public opinion orientation of new media and using 3S technology to help the government make emergency response and command for public health emergencies.

RETRACTED

With the rapid development of network information technology, a large number of new media and self-media have emerged. As an important medium for information semination, media has the characteristics of fast dissemination and wide dissemination. In addition, due to the wide audience, the information disseminated by the media will seriously affect the judgment and choice of the public, and the fast-developing of network information technology now makes the public understand information very quickly and timely.

Traditional media mainly include newspapers and magazines, TV broadcasts, and mobile phone text messages. When a public health emergency occurs, the public will obtain the news and information they want through a variety of channels. According to the results of the questionnaire survey, the public generally obtains information on public health emergencies through the Internet channels such as Weibo, WeChat official account platform, TikTok short video, news network, and other traditional media such as newspapers and magazines, television, radio, and some other media.

Table 1 shows that the public's access to information in public health emergencies in each year is different. When the SARS outbreak occurred in 2003, because new media such as Weibo, WeChat, and TikTok had not yet appeared, the sources of information obtained by the people mainly rely on traditional media such as newspapers, magazines, and television broadcasting. Among them, television broadcasting is the main source of information obtained by the people, accounting for 59.23%, followed by newspapers and magazines, accounting for 14.75%. In addition, QQ social software is also obtained by people. One of the important channels for SARS information, accounting for 14.3%; when the H1N1 avian flu occurred in 2009, Weibo, WeChat, and other software began to rise, and a small number of users relied on it to obtain H1N1-related reports and information. Secondly, the proportion of obtaining news through QQ and news networks has increased, accounting for 23.65% and 11.58%, respectively. The proportion of newspapers and magazines has dropped to 11.58%; and in 2020, with the further development of new Internet media, Weibo and WeChat platforms have developed and improved rapidly, and the emergence of TikTok short videos has further broadened the channels for the public to obtain epidemic information. At this time, we can see that the main channels for the public to obtain news about the COVID-19 virus are Weibo, WeChat, and TikTok, which together account for 91.51% of the total. It can be seen that new media for obtaining information on public health emergencies have an absolute advantage.

RETRACTED

### 3.2. Flowchart of Multimodal Corpus Construction

The emergency corpus has its own characteristics, construction methods, and processes in construction. We need to consider from the basic principles of construction, corpus sources and acquisition methods, corpus storage format and language material processing, and other aspects. We design the following flowchart of multimodal corpus construction as shown in Figure 2.

### 3.3. Steps of MACPHE

This article makes a comprehensive analysis based on the types of public emergencies in reality and the characteristics of news language materials and proposes the following classification steps:

1. Raw data process and input

After installing ELAN6.4 version on the computer side, then installing VLC media. The video that needs to be analyzed is converted to wav format file by VLC media player key. Finally, save audio and video files in the same folder.

(2) Segmentation and annotation

The segmentation and annotation of multimodal public health emergency corpus is the core part of the construction of the corpus. Based on the needs and purposes of the study, taking the daily COVID-19 newsletter video released by CCTV as an example, the focus of the study is on the speaker's discourse and journalists‘ questions.

(3) Multimodal data classification and terminology collection

By summarizing the relevant multimodal emergency corpus and retrieving different data sets, the researchers obtained the frequency of a certain public health disease at a certain stage and grasped the potential public health emergency situation at home and abroad in this period. Furthermore, collect the key terminology.

### 3.4. Public Health Multimodal Corpus for Further Processing

Before further processing of the corpus, we established maintainable term bases for natural disasters, accidents, public health events, and social security events and established user-defined dictionaries for word segmentation. In order to use the corpus more accurately, if the terminology changes, such as the country naming “coronavirus disease,” we will not only maintain the terminology database and custom dictionary but will also include the “COVID-19” sentence from the deep processing.

According to the four types of the corpus, different processing methods are adopted. For short text corpora, we only store its raw corpus (focusing on extracting emoticons with rich meaning). For texts of laws and regulations, we perform word segmentation processing and store raw corpus and word segmentation data. News event like text corpus processing way, for event extraction and visualization (emergency language service event annotation visualization processing, the author has a separate article), etc., we will carry out word segmentation tagging part of speech, syntactic tagging and semantic tagging, and store it into the database.

RETRACTED

There are four storage methods for corpus, part-of-speech tagging corpus, syntactic tagging corpus, and semantic tagging corpus. For images corpus, we apply search engine to access official website of WHO, and some national public health websites.

As it is shown in Figure 3, multimodal (MM hereafter) corpus generally presents “data” in four different modes, as spoken (audio), video, image, and textual records of real-life interactions, accurately aligning within a functional, search-able corpus setting [21]. From the existing multimodal corpus, the major modal is textual data, accounting for more than 75%, the second modal is video data accounting for 15%, and the rest of the raw data come from audio and image modal.

## 4. The Research Model

The major three sources of multimodal corpus are National Health Commission of the P.R.C Website(http://www.nhc.gov.cn/), WHO website, and some official video channels, such as Xuexi channel and CCTV channels.

### 4.1. Multimodal Aligned Corpus Processing Tools: ELAN

ELAN (EUDICO Linguistic Annotator) is an annotation tool that allows you to create, edit, visualize, and search annotations for video and audio data. It was developed at the Max Planck Institute for Psycholinguistics, Nijmegen, The Netherlands, with the aim to provide a sound technological basis for the annotation and exploitation of multimedia recordings. ELAN is specifically designed for the analysis of language, sign language, and gesture, but it can be used by everybody who works with media corpora, i.e., with video and/or audio data, for purposes of annotation, analysis, and documentation.

ELAN as a free technical tool can be downloaded from the following website (https://archive.mpi.nl/tla/elan/download). As shown in Figure 3, ELAN supports speech and/or video signals, together with their annotations; time linking of annotations to media streams; linking of annotations to other annotations; unlimited number of annotation tiers as defined by the users; different character sets; export as tab-delimited text files; import and export between ELAN and Shoebo [22].

It can be seen from Figure 4 that it is possible to match up arbitrary pieces of text (annotations) with sections of audio or video (media), producing documents (transcripts) which permits fluid navigation between text and media of public health emergencies. With ELAN, a user can add an unlimited number of textual annotations to audio and/or video recordings. An annotation can be a sentence, word or gloss, a comment, translation, or a description of any feature observed in the media. Annotations can be created on multiple layers, called tiers. Tiers can be hierarchically interconnected. An annotation can either be time-aligned to the media or it can refer to other existing annotations. The content of annotations consists of Unicode text and annotation documents are stored in an XML format (EAF).

RETRACTED

### 4.2. Syntax Annotation, Semantic Role Annotation, and Manual Proofreading

With the in-depth development of language technology and corpus technology, researchers are no longer satisfied with obtaining intuitive language facts from the corpus. Syntax annotation and semantic role annotation map the shallow vocabulary and part-of-speech information to the tree structure of each component of the sentence. In the era of deep learning, its application in NLP is continuously deepened, especially the LSTM model that carries the syntactic relationship, the CNN model, and the BERT model that carries the position information of the sentence, which makes the complex and difficult work of syntactic labeling and semantic role labeling. It seems less important. However, the corpus that has been marked by syntax and semantic roles has extremely high value and broad prospects, especially in the research and practice of linguistics and natural language processing.

### 4.3. Corpus Information Fields and Storage Format

The field design and storage format of the corpus determine the purpose and scalability of the constructed corpus. Extensible Markup Language (XML) is a markup language that provides a data description format. The language spans multiple platforms, enabling more accurate content declarations and more meaningful search results. In addition, XML separates data from presentation and processing and is highly extensible.

Before storage, we will perform sentence processing on all texts. XML schema is defined as the following table. The storage adopts UTF-8 encoding format. There are two main elements in the XML document, article Info and text. <articleInfo> records external information of the corpus, including title, time, source, category, subject matter, and author. <text> is the main text, recording paragraph information, sentence information, raw corpus in units of sentences, part-of-speech tagging corpus, dependent syntactic tagging corpus, and semantic role tagging corpus. The steps required are shown in Table 2.

## 5. Discussion

This thesis carries out a multimodal discourse analysis of the construction and application of MACPHE. Based on a multimodal corpus, the present study aims to gain insight in the construction relationship between sports industry development and health emergency service. From the perspective of big data, this paper takes the impact of the construction of public sports health emergency corpus as a research topic, which is innovative and conforms to the current research direction. The primary finding of this study is to ascertain the ways in which multimodes are interrelated to construct meaning of public health emergency events in multimodal contexts, and to further explore their contributions to the strategy-making process. In addition, the study also explored the influence of social media and big data on the realization of MACPHE modes.

RETRACTED

Through the in-depth study of public health emergency in the field of multimodal corpus, the study has provided further evidence confirming the realization of MACPHE modes. The study reveals that the analysis of modal density, which encompasses modal complexity and modal intensity, can be used to mirror the multiple modes in strategy-making. Therefore, careful analysis is required to explore the meaning of different semiotic sources in multimodal of public health emergency corpus. The most obvious limitation in this research is the small sample size and the small number of multimodal modes, which is limited to the repentance of the raw data. If more data can be collected and annotated with more modes, the multimodal analysis can be conducted with sounder statistics.

## 6. Conclusion

This article reviews the origin, definition, and composition of national and foreign language proficiency concepts and multimodal corpus at home and abroad, discusses the significance and principles of emergency corpus construction, and proposes a technical route and process for constructing public health emergency corpus construction. We believe that national language ability is built on big data resources, corpus systems, and natural language process operations and is divided into internal ability and external use; national language ability resources include language resources and language-related talents, of which the accumulation and development of language resources and language technology are also basic factors that should not be ignored. It is worthy of research and discussion in academia to promote the construction and development of Chinese language strategy and planning theory. In the future, we will develop more efficient algorithms and more affluent corpus for detecting public health problems and natural disasters based on the National Emergency Corpus (NEC) [23].

## Figures and Tables

**Figure 1:** Architecture and classification of emergency corpus for public health emergency.

RETRACTED

**Figure 2:** Flowchart of multimodal corpus construction.

**Figure 3:** Classification of multimodal corpus.

**Figure 4:** Official download website of ELAN.

**Table 1:** Major channels to obtain public health emergencies from media.

Public health emergency	Weibo	WeChat	QQ	TikTok	News site	Newspapers and magazines	TV broadcast
SARS	0%	0%	14.3%	0%	9.63%	14.75%	61.32%
H1N1	0.63%	1.48%	23.65	0%	11.58%	52.14%	0%
COVID-19	43.67	23.16%	4.15%	35.68%	2.37%	1.03%	4.69%

**Table 2:** Definition and raw data processing of XML schema.

Code NO.	Description of the date processing
001	<?xml version=“1.0” encoding=“UTF-8”?>
002	<xs:schemaxmlns:xs=“http://http://www.w3.org/2001/XMLSchema”
003	targetNamespace = “http://www.w3schools.com”
004	xmlns=“http://www.w3schools.com” elementFormDefault=“qualified”>
005	<xs:element name=“articleInfo”
006	<xs:complexType>
007	<xs:sequence>
008	<xs:element name=“title” type=“xs:string”/>
009	<xs:element name=“time” type=“xs:string”/>
010	<xs:element name=“source” type=“xs:string”/>
011	<xs:element name=“author” type=“xs:string”/>
012	<xs:element name=“classify” type=“xs:string”/>
013	<xs:element name=“theme” type=“xs:string”/>
014	</xs:sequence>
015	</xs:complexType>
016	</xs:element>
017	<xs:element name=“text”>
018	<xs:complexType>
019	<xs:sequence>
020	<xs:element name=“sectID” type=“xs:string”/>
021	<xs:element name=“sentenceID” type=“xs:string”/>
022	<xs:element name=“sentence” type=“xs:string”/>
023	<xs:element name=“sentenceCut” type=“xs:string”/>
024	<xs:element name=“sentenceDependency” type=“xs:string”/>
025	<xs:element name=“sentenceSemantic” type=“xs:string”/>
026	</xs:sequence>
027	</xs:complexType>
028	</xs:element>
029	</xs:schema>

## Data Availability

The data used to support the findings of this study are available from the corresponding author upon request.
